The article "What is policy content and how is the public's policy support? A policy cognition study based on natural language processing and social psychology" was published in 2022. Journal: Front Psychol.

# What is policy content and how is the public's policy support? A policy cognition study based on natural language processing and social psychology

**DOI:** 10.3389/fpsyg.2022.941762

**Published:** 2022-10-04

**Authors:** Lingyi Zhou, Dingzhang Dai, Junxia Ren, Xiaoxu Chen, Siming Chen

**Affiliations:** ^1^School of International Relations and Public Affairs, Fudan University, Shanghai, China; ^2^School of Data Science, Fudan University, Shanghai, China; ^3^Tiandao Fintech Co., Ltd., Hangzhou, China; ^4^Zhelixin Co., Ltd., Hangzhou, China

**Keywords:** policy cognition, policy support, policy content, natural language processing, social psychology

## Abstract

Public policy plays a critical role in coordinating social resources, providing public services, and promoting public value. However, few studies have systematically investigated the public's policy cognition from the objective aspect of policy content and the subjective aspect of target audience's policy support. To fill this gap, we explore the policy content via natural language processing and also policy support from the perspective of social psychology. Specifically, regarding the policy content analysis, we collect over one thousand policy documents and design an annotation system by analyzing the policy content, basic structure and text features, and then utilize text classification and information retrieval models based on the Chinese large-scale pre-trained models. Moreover, according to the policy tools identified in the content analysis, our paper investigates the audience's policy support for these tools and its influential factors. Based on a sample of 476 respondents from the whole country, we adopt the ordinary least square method to explore the key factors of policy support for supply, demand and environmental tools from three variables: political trust, policy effectiveness and knowledge of policies. This study contributes to existing literature by forming a structured understanding of policies and exploring public support for policy tools, which could benefit the practitioners during the policy-making process and also enhance successfully policy implementation.

## 1. Introduction

The government plays a critical and decisive role in promoting economic development, offering social services and improving citizens' living standards in China. Generally, governments at all levels would launch a large number of public policies to allocate limited resources, solve social problems and pursue public value. And the public would generate their cognition of policies, which is vital to both policy-making and also implementation. Cognition are thoughts, awareness, perceptions, attitudes, and beliefs (Newell, 1990), involving social constructions of reality (Berger and Luckmann, 2016). Most studies about policy cognition have explored its role in the public's behaviors or cognitive appraisals based on the theories of planned behavior (Ajzen, 1991), cognitive behavior (Allen, 2018), cognitive evaluation (Wang et al., 2020), and others. Some scholars constructed a cognitive model that implementing agents' policy sense-making is a function of the interaction of policy signals, agents' knowledge, beliefs and experience and also the circumstances or context (Spillane et al., 2002). Existing literature mainly studies policy cognition from a subjective perspective. However, we argue that the objective components of policy texts are also the constituting elements during the cognitive process. Therefore, in this paper, we develop a more comprehensive definition of policy cognition as individuals' sense-making from and about policies objectively and subjectively. From the objective aspect, the composition of policy documents represents ideas about reforming practice and also the messages sent to the implementing agents and the target audience. From the subjective aspect, multiple interpretations of a single policy might exist due to individuals' beliefs, values, emotions and also the situation or context based on the work in social psychology. Additionally, the composition or content of policy texts are the objects of individuals' subjective cognition. Thus, linking the objective and subjective aspects of policy cognition is beneficial to the all-round understanding of policies and also providing suggestions on policy design to practitioners. Policy support is one of the most important dimensions of the subjective cognition, and we would focus on it in this paper. According to data published by the Zhejiang Provincial People's Government^1^, over two thousand policy documents are released each year in Zhejiang, covering various policy areas as economic development, industry planning, traffic construction, social security and others. For better understanding the public's cognition of policies, our research tries to investigate it from both objective and subjective perspectives, systematically exploring the content of policies and the audience's support level toward them respectively.

The article "What is policy content and how is the public's policy support? A policy cognition study based on natural language processing and social psychology" was published in 2022. Journal: Front Psychol.

First, from the objective aspect, what is the content of public policies? With the development of big data era and the disclosure of government information, many scholars have started to use natural language processing techniques for deep text mining of public policies (Spruit and Ferati, 2020). Recently, many machine learning and deep learning models have been constructed to accurately extract specific factual information from natural language text and classify large amounts of textual content automatically (Kowsari et al., 2017; Ansari et al., 2018). The extracted information, including entities, relationships, events, etc., plays an important role in downstream tasks and application scenarios, like machine translation, question answering system. Actually, the text structure of policy documents is clearly delineated and words have a unified standard usage. Thus, it would be efficient and effective to analyze policy text by employing natural language processing techniques. However, there are some limitations in existing literature. Some studies adopt the unsupervised learning-based approach, which might challenge the validation of the method and the stability of model due to the absence of a gold standard and scholars' subjective judgments (Wilkerson and Casas, 2017). Other studies employ the supervised learning, but they haven't fully integrated the machine learning model with policy elements from domain experts' perspective, and the systematic analysis of the content of Chinese policy documents is still lacking (Schoonvelde et al., 2019). To fill these gaps, we construct a comprehensive policy label system to systematically summarize the various elements of policy documents with the collaboration between public administration researchers and computer science researchers. Then, we analyze the text of policy documents through machine learning and deep learning models based on large-scale Chinese pre-trained models, to understand policy content.

Second, from the subjective aspect, to what extend does the audience support these policies? Policy support represents the legitimacy of policy design, and also plays a critical role in successfully policy-making and implementation. In China, the governments have standardized the procedure for online consultation since 2008 and made substantial efforts to include the general public into policymaking processes (Balla, 2017; Kornreich, 2019). However, existing literature on policy content analysis has paid less attention to the level and formation process of policy audience' support. Regarding the literature of policy support, scholars have explored the effects of political trust, perceived fairness, perception of costs, perceived risk, and knowledge (Eriksson et al., 2006; Zannakis et al., 2015; Zhou and Dai, 2017). But the formation mechanism of policy support for multiple policy tools is absent. Specifically, supply, demand and environmental tools have been identified in text analysis, thus, our paper investigates the audience's support for these tools and its influential factors from the perspective of social psychology. Based on a sample of 476 respondents from the whole country, we adopt the ordinary least square method to explore the key factors of policy support for supply, demand and environmental tools from three variables: political trust, policy effectiveness and knowledge of policies.

The article "What is policy content and how is the public's policy support? A policy cognition study based on natural language processing and social psychology" was published in 2022. Journal: Front Psychol.

The rest of this paper is organized as follows. Section 2 presents the literature review. Section 3 introduces the methodology and provides results of model analysis. Section 4 presents a further discussion and conclusion.

## 2. Literature review

Since the policy document has a distinct structure and similar wording, its parsing can be naturally converted into several natural language processing tasks, which provides us with an objective understanding of policy cognition. Based on the accurate classification of elements in policy documents, we could analyze the policy text automatically through natural language processing technology, to gain a better understanding of policy information. Additionally, policy support is a key factor of policy legitimacy and successful implementation, also delineating the subjective understanding of policy cognition. In this section, we summarize both the literature of policy content analysis and policy support.

### 2.1. The literature on policy content analysis

#### 2.1.1. Automated political text analysis

Text is pervasive and persistent artifact of political behavior (Monroe and Schrodt, 2017). With the development of the Internet, researchers have access to much more data than ever before, and text-as-data research has gradually become the mainstream in political science (Wilkerson and Casas, 2017). However, the cost of manually analyzing large scale unstructured text data is unaffordable. Automated text analytics could solve this problem and has been developed in both political science and political psychology research, but there are still many interdisciplinary research questions left for further exploration (Schoonvelde et al., 2019).

Existing political text analysis methods are mostly quantitative and statistic based. These methods require the researcher to specify which elements of the document are used to construct text features, such as studying the dynamics of parliament by examining the frequency of specific words at different times (Eggers and Spirling, 2018). Regarding machine learning-based political text analysis, scholars are usually more concerned with the output of the model. For example, based on topic or scaling models, unsupervised machine learning methods such as K-means, PCA, LDA, etc., are adopted to learn thematic content and policy position from text; or documents are first manually coded into predefined categories and then used to train models to classify documents into known categories (Grimmer and Stewart, 2013). Natural language processing techniques expand the scope of this research in a lot of recent research, such as automatically extracting special parts from the document and tag different references to the same entity (Wilkerson and Casas, 2017) or isolating substantive content from the document (Denny et al., 2015).

The article "What is policy content and how is the public's policy support? A policy cognition study based on natural language processing and social psychology" was published in 2022. Journal: Front Psychol.

Deep learning has been well used in many fields recently, but natural language processing techniques based on deep learning have not been widely adopted in automated policy text analysis (Schoonvelde et al., 2019). Therefore, this paper uses multiple deep learning models in two NLP tasks for policy content analysis, thereby attempting to achieve automated analysis at a deeper semantic level.

#### 2.1.2. Text classification

Text classification refers to labeling a given sentence, paragraph or article with the corresponding category. Before 2010, text classification adopted generally classical machine learning models based on statistics, such as TF-IDF (Yun-tao et al., 2005), naive Bayesian (Maron and Kuhns, 1960), SVM (Joachims, 1998), and random forest (Breiman, 2001).

Since Word2Vec (Mikolov et al., 2013) was proposed in 2013, the application of deep learning in the field of NLP has developed rapidly. The advanced text classification methods are usually based on deep learning neural network models. Convolutional Neural Networks (CNNs) are widely used networks that contain convolutional filters capable of extracting picture features, so they were first applied to picture classification tasks. Kim (2014) applied CNN to sentence classification and proposed TextCNN, which performed considerably well and showed that unsupervised pre-training of word vectors is essential for deep learning in NLP.

In addition, Recurrent Neural Networks (RNNs) are also widely used in NLP. Their unique sequence processing is very similar to the way humans read, which can effectively learn location information in the text. In recent years, there are many studies on RNNs for text classification tasks. Liu et al. (2016) studied RNN text classification based on multi-task learning, and Dieng et al. (2016) proposed a RNN with long-range semantic dependencies. However, it should be noted that RNNs may have a gradient disappearance during backpropagation. To solve this problem, Long Short-Term Memory (LSTM) uses three gates to selectively forget and remember information, which enables it to learn long-term dependencies (Graves, 2012).

In 2015, Bahdanau et al. (2014) first proposed the “Attention” mechanism. Inspired by them, many researchers started to apply the attention mechanism to text classification tasks. Google proposed the large-scale pre-trained model BERT (Devlin et al., 2019), which has shown remarkable text representation ability. This language model has achieved outstanding results in text classification tasks (Sun et al., 2019).

The article "What is policy content and how is the public's policy support? A policy cognition study based on natural language processing and social psychology" was published in 2022. Journal: Front Psychol.

Text classification is one of the most fundamental tasks in natural language processing, and classifying texts enables the conversion of unstructured data into categorical data, which can be used to analyze text structure from holistic perspective. Therefore, this paper tries to train models for policy sentence classification on a sufficient number of policy texts to achieve a more systematic understanding of policies by using machine learning and deep learning techniques under a self-designed labeling system.

#### 2.1.3. Named entity recognition

Named Entity Recognition (NER) aims to find the boundaries of entities in texts and classify them into pre-defined classes. Collobert et al. (2011) used neural networks in NER and proposed two network structures, namely window approach and the sentence approach. After that, more and more studies have combined neural networks with traditional statistical machine learning methods, and a representative model is BiLSTM-CRF (Huang et al., 2015). It uses a bidirectional Long Short-Term Memory (Bi-LSTM) network and conditional random field (CRF) to solve the text annotation problem, which is still one of the mainstream methods for named entity recognition. Based on this model, Liu et al. (2018) further added a character-level language model for training, which tends to be more effective.

Furthermore, the Attention mechanism has also been applied to the named entity recognition task. Rei et al. (2016) used both character- and word-level embedding in the framework of sequence annotation, and dynamically decide how much information to use from a character- or word-level component by adopting an attention mechanism. After Google proposed the BERT (Devlin et al., 2019) model, named entity recognition was also regarded as a downstream task. The BERT-BiLSTM-CRF is one of the excellent models for NER. This model was also widely used in the Chinese NER task, for example, Dai et al. (2019) applied the model to Chinese electronic health records named entity recognition and achieved optimal results in the test models.

In recent years, many improved methods have also been applied to the Chinese and English NER tasks, significantly promoting the results. Li et al. (2020) solved the problem of lexical loss in lattice-LSTM and used relative position encoding to make Transformer adapt to NER. Wu et al. (2021) proposed a two-stream model capable of combining character features, word features and radical features. Yan et al. (2019) improved the Transformer so that it can capture the distance and direction information between tokens. Li et al. (2021) proposed a unified model of NER, W2NER, using a unified Word-Pair tagging approach to model different types of NER tasks.

The article "What is policy content and how is the public's policy support? A policy cognition study based on natural language processing and social psychology" was published in 2022. Journal: Front Psychol.

Named entity recognition is the basis for many natural language processing tasks, and deep learning methods have been well-applied to these tasks. However, the domain adaptation of these techniques is often challenging and lacking. Therefore, we design and compare several deep learning models to retrieve policy information entities based on the characteristics of policy documents.

### 2.2. The literature on policy support

#### 2.2.1. Policy support and its influential factors

Policy support represents the legitimacy of policy design, which is vital to effective policy design (Fung, 2006). Legitimacy is used as an overall term for the degree to which a certain policy is accepted by the citizens (Woodside, 1998). Policy makers are supposed to pay enough attention to the characteristics of the target audience, including their attitudes, behaviors, motivations and previous reactions to policy initiatives directed at them (Bagchus, 1998; Bemelmans-Videc et al., 1998a; Egmond et al., 2006). Previous research has showed various factors would influence public attitude toward policies or regulations, such as perceived fairness (Jakobsson et al., 2000; Jagers et al., 2010; Zannakis et al., 2015), perceived policy effectiveness (Chen and Zhao, 2013), policy characteristics (De Groot and Schuitema, 2012), psychological factors (Eriksson et al., 2006), trust in authorities (Bronfman et al., 2008; Jagers et al., 2010; Zannakis et al., 2015; Zhou and Dai, 2020), ideology (Jagers et al., 2010), and so on. In this research, we try to investigate the roles of political trust, policy effectiveness and knowledge of policies in policy support.

Specifically, both political trust and policy effectiveness have positive effects on both people's attitude toward government regulation and the level of compliance (Jagers and Hammar, 2009; Harring and Jagers, 2013; Zannakis et al., 2015). The audience tends to support for policies those are more effective or made by the authorities they have a high level of trust in. Knowledge is crucial to people's attitudes toward policy, both the amount and accuracy (Zhou and Dai, 2017). Some scholars have stated knowledge is an antecedent to individual's attitude or value (Kollmuss and Agyeman, 2002; Bamberg and Möser, 2007). And we believe that knowledge of policies has positive effects on the audience's support level as they would know more benefits of these polices.

The article "What is policy content and how is the public's policy support? A policy cognition study based on natural language processing and social psychology" was published in 2022. Journal: Front Psychol.

#### 2.2.2. Policy support for different policy tools

The target audience's policy support varies via different policy tools. Policy tool, is the specific instrument adopted to achieve policy goal. There are different types of policy tools, such as regulation and economic means (Linder and Peters, 1989; Bemelmans-Videc et al., 1998b; Goulder and Parry, 2020), and supply, demand, and environmental instruments (Rothwell and Zegveld, 1981). As there are many differences among alternative policy tool types, such as the degree of coercive power, the distribution and visibility of cost burden, the uncertainty about goal achievement and others (Hahn and Stavins, 1991; Stavins, 1998). The audience may generate different levels of support for these policy tools (Loukopoulos et al., 2005), but this difference has seldom been mentioned in previous studies. To bridge the literature gap, we focus on public support towards different types of policy instruments in this research.

Although there are different categorizations of policy tools, the classification developed by Rothwell and Zegveld (1981) is rooted in evaluating industrial policies and science and technology policies, which is consistent with the policy field of our research. So we adopt this widely used classification including supply, demand and environmental instruments. Supply tools refer to provision of financial, manpower and technical assistance, supporting the enterprises with necessary resources or infrastructure. Demand tools include central and local government purchases and contracts, aiming at strengthening enterprise survival and success. At last, environmental tools mean that the government provides favorable environment in which enterprises operate, such as taxation policy, patent policy, and regulations. In this paper, we would investigate the target audience's preference and support level of supply, demand and environmental policies, and also compare the differences of influential factors among these tools.

## 3. Methodology

According to the research questions, our paper contains two parts, namely, policy text and policy support analysis, which demonstrates policy cognition from objective and subjective aspects respectively. On the one hand, we try to achieve a more structured understanding of the policy text by classifying sentences in policy documents and retrieving the essential information in them under a comprehensive policy label system. On the other hand, this research investigates the effects of political trust, policy effectiveness and knowledge on policy support of different tools. The main structure of this paper is shown in Figure 1.

The article "What is policy content and how is the public's policy support? A policy cognition study based on natural language processing and social psychology" was published in 2022. Journal: Front Psychol.

**Figure 1:** Main structure of this paper.

### 3.1. Policy content analysis

#### 3.1.1. Pre-analysis

The data for policy content analysis were obtained from relevant government departments in Zhejiang Province, including the Development and Reform Bureau, the Administration for Market Regulation Bureau, the Human Resources and Social Security Bureau and others. We collected 2,899 original published policy documents, wherein the text of 1,481 documents was extractable, and finally obtained the text of 1,325 documents after cleaning and de-duplicating. To get a prior understanding of our dataset, we randomly selected 81 documents for pre-analysis. After segmenting these documents according to the stop words, the structural features of the text paragraphs and special textual content, we performed a statistical analysis based on the relevant literature of social science and natural language processing. We found some characteristics of the Chinese policy texts in our data: Firstly, the text structure can be divided very clearly and the category of each sentence is obvious, which is highly related to the types of context and their positions in the text. For example, we counted the position of several policy elements *via* dividing the serial number of relevant sentences by the total number of sentences in the document. As shown in Figure 2, the content related to policy tools tends to appear consecutively in the middle and later parts of the document, while the content related to policy goals appears more often at the beginning of the document. Secondly, the policy text explicitly contains information that can be extracted structurally, such as the validity period, the implementing department, and other basic information of a specific policy. And there are long sentences and entities in the text as shown in Figure 3, which poses a challenge for our extraction. Due to these characteristics, this paper explored the text analysis of policy documents through policy sentence classification and policy information retrieval, and designed the methods used in the task based on the characteristics.

**Figure 2:** The position of several policy elements.

**Figure 3:** Length distribution of sentences containing policy entities and length distribution of policy entities in 81 documents.

In order to assess the feasibility of classifying the texts of policy documents, we observed whether there is a possibility that these texts can be classified. We extracted some important and representative keywords from the text data of 30 policy documents. For discovering their commonalities and unique characteristics, we performed network visualization based on their common occurrences. As shown in Figure 4, the pink nodes are extracted keywords and gray nodes are policy documents. If one document contains a keyword, the gray node indicating this document has a link to the corresponding pink node. The size of the pink nodes indicates how many times these keywords are mentioned in multiple documents. It can be clearly seen that the nodes in the figure have a tendency to aggregate in clusters, and the keywords contained in such clusters all have similar words and meanings, which indicates that there is a clear typological distinction among the texts of policy documents and this distinction can be expressed in its content.

The article "What is policy content and how is the public's policy support? A policy cognition study based on natural language processing and social psychology" was published in 2022. Journal: Front Psychol.

**Figure 4:** Network visualization of co-occurrences of key words in policy texts.

For example, we can see “incentive”, “subsidy” are the most mentioned words in the policy text. We can also see that the document 6 and 16 are similar, as they both mentioned “province”, “innovation,” and “incentive”. Through the visualization we can have an overview understanding of the data.

According to the above pre-analysis, we decided to carry out the policy content analysis in two tasks, namely, sentence classification and information retrieval. Then we need to identify the elements of policy documents as labels for these two tasks. Based on the theory of policy tools in policy studies (Rothwell and Zegveld, 1981; Linder and Peters, 1989; Bemelmans-Videc et al., 1998b; Goulder and Parry, 2020) and some common information related to policy documents, we summarized the following elements for policy texts and used them in the tasks of policy content analysis in this paper.

The content of policy documents can be classified into the following elements.

• **Policy goal**: The objectives the government is seeking to achieve.
• **Application review procedure**: All matters related to application and audit, such as application procedures, materials required for application, audit procedures, etc.
• **Funds management**: All matters related to funds management, including sources of funds and management rules.
• **Supervision and evaluation**: All matters related to the regulatory or evaluation tools employed by the government for ensuring policy implementation, including monitoring and assessment.
• **Policy tools—Supply tools**: The policy tools aim at directly increasing the supply of enterprises through the provision of financial, manpower and technical assistance. These tools can be divided into specific categories of personal training (personnel training plan, the education and training systems, etc.), funding support (R&D funds and infrastructure development funds, etc.), technical support (technical consultation and technical infrastructure construction, etc.) and public services (supporting facilities and policy environment, etc.).
• **Policy tools—Demand tools**: Policy tools aim at reducing market uncertainty and increasing the likelihood of enterprise success. These tools include government procurement, public-private partnerships (joint investment, joint technical research, joint development planning, etc.), and overseas partnerships (introducing foreign capital; cooperation with overseas governments, enterprises or research institutions, etc.).
• **Policy tools—Environmental tools**: The policy tools aim at providing a favorable environment for enterprises through tax, financial, and regulatory policies to indirectly promote their innovative activities. These policy tools can be divided into more specific categories, including regulation (regulations and standards of market supervision), object programming (top-level planning), tax breaks (tax deductions and refunds to support enterprise development, including investment deductions, accelerated depreciation, tax exemptions and rental tax deductions, etc.), financial support (loans, subsidies, venture capital, credit guaranties, funds, risk control, and other financial support to enterprises through financial institutions), organizational building (setting up organizations or team building for leadership, supervision and service), policy advocacy (publicizing relevant policies for industrial development).

The article "What is policy content and how is the public's policy support? A policy cognition study based on natural language processing and social psychology" was published in 2022. Journal: Front Psychol.

Regarding the common information of policy documents, the following elements can be defined.

• **Policy name**: Full name of the policy.
• **Policy document number**: It is the sequential number of the total number of policy documents issued by the government in a given year. Its basic structure includes the words representing the issuing authority, the year code and the serial number of the issuing document.
• **Issuting area**: The cities where the government issues this policy.
• **Policy-making department**: The governmental department that formulated the policy and issued it.
• **Policy implementation department**: The governmental department that responsible for implementing the policy.
• **Validity period**: The period the policy remains valid.

These elements can be the basis for further policy content analysis.

#### 3.1.2. Policy sentence classification

##### 3.1.2.1. Task description

Based on the overview through pre-analysis, this task aims to classify the sliced sentences after cutting the policy texts. Our automated policy sentence classification model enables efficient classification of a large number of policy document texts, thus helping to analyze the structure and composition of policy text content more quickly and accurately, and also helping the government and related personnel to interpret policy texts. The categories are labeled by the elements of policy content mentioned above, including: policy goal, application review procedure, funds management, supervision and evaluation, policy tools—supply tools, policy tools—demand tools, policy tools—environmental tools.

The article "What is policy content and how is the public's policy support? A policy cognition study based on natural language processing and social psychology" was published in 2022. Journal: Front Psychol.

Specifically, policy sentence classification is modeled as a text classification task in natural language processing. Text classification refers to mapping a piece of text containing information to a given class or classes. In this paper, the classification process refers to doing multiple classifications of policy texts at the sentence level. Since policy texts contain complex contents and longer sentences, we address this task by comparing various machine learning-based and deep learning-based approaches to classify policy sentences.

For this task, our approach is to use a Chinese pre-trained model to obtain a vector representation of features for sentences, and then use machine learning-based and deep learning-based models to classify the sentences.

##### 3.1.2.2. Distributed representation

First, we need the representation of the policy text for the classification model. Previous approaches to NLP tasks using statistical machine learning have often relied on feature engineering designed by experts based on a priori knowledge. High-quality feature engineering contributes significantly to model effectiveness, but at the same time sacrifices model generality. In deep learning-based approaches, the simplest features are non-distributed representations, such as one-hot vectors, which are usually very sparse, inefficient, and can cause dimensional catastrophes. The other feature is distributed representation, which maps the semantics or features of texts to neurons. It ensures that there is discrimination between the features corresponding to different neurons, thus obtaining a low-dimensional and dense vector to characterize the text. This vector represents the features extracted by neural network, and is the most common representation of text data for natural language processing.

In this task, we use a word vector obtained by Word2vec, which is pre-trained on a large comprehensive domain corpus using a skip-gram model with negative sampling methods (Li et al., 2018), and no parameters related to the distributed representation are needed in our training.

##### 3.1.2.3. Machine learning models

Although machine learning models usually have simple structures and the parameters are relatively few, these models tend to perform well in complex tasks with good domain adaptation. In the machine learning models we used, for a given sentence, after obtaining the word vector by feature engineering based on Word2Vec, the vector representation of all words (300 dimensions) is averaged in each dimension, and then it is spliced with the length of the sentence and its position in the text (serial number of the sentence in the file / total number of sentences in the document) to get a 302-dimensional vector as the representation of this sentence.

The article "What is policy content and how is the public's policy support? A policy cognition study based on natural language processing and social psychology" was published in 2022. Journal: Front Psychol.

We use Support Vector Machine (SVM) and eXtreme Gradient Boosting (XGBoost) (Chen and Guestrin, 2016) as the classifiers. The basic model of SVM is the linear classifier with maximum interval defined on the feature space. Its basic idea is to solve for the separated hyperplane that can correctly partition the training data set and has the maximum geometric interval. In our model, a one-vs-one scheme is used to handle multiclass support. The decision function of SVM is shown in the following equation.


(1) $$\begin{array}{l} f\left(x\right)=sign\left(w^{*}\cdot x+b^{*}\right) \end{array}$$

where *x* is the vector representation of the sentence, *f*(*x*) is the label predicted by the model, w^*^ and b^*^ are the optimal parameters determined by only a few support vectors, which makes the model both simple and relatively robust.

XGBoost is an optimized algorithm based on Gradient-Boosted Decision Trees (GBDT), which is an additive model composed of multiple base models. The decision function of XGBoost is as follows.


(2) $$\begin{array}{l} f\left(x\right)=\overset{k}{\underset{t=1}{\sum }}f_{t}\left(x\right) \end{array}$$

where *x* and *f*(*x*) are defined in the same way as SVM, and *f*_*t*_ denotes the basic model that makes up XGBoost. With this ensemble learning strategy, XGBoost has the advantages of high accuracy, support for parallelism, and more flexibility, and is a commonly used model in supervised learning.

##### 3.1.2.4. Deep learning models

One of the advantages of deep learning models is that they are end-to-end, which avoids inconsistencies in training objectives and the accumulation of errors across modules in multi-step models. The deep learning classification models we employed include TextCNN and BiLSTM-Attention, both of which are commonly used supervised learning classification models.

TextCNN (Kim, 2014) consists of only one convolutional layer, one max-pooling layer, and one output layer for multi-classification using the softmax activation function. In the convolutional layer, three convolutional kernels of sizes 3, 4, and 5 are used to extract features from distributed word vectors. Since TextCNN is a simple structured neural network with a small number of parameters and computation, it has a fast training speed while ensuring the correct rate.

The article "What is policy content and how is the public's policy support? A policy cognition study based on natural language processing and social psychology" was published in 2022. Journal: Front Psychol.

The BiLSTM-Attention (Zhou et al., 2016) model adds the attention mechanism to the BiLSTM (Huang et al., 2015) model. LSTM differs from the way CNN extracts text features spatially; it extracts them temporally, which is closer to the way humans think. Compared with LSTM, Bi-LSTM can better capture the contextual information in the sentence, and the Attention mechanism can get better interpretability and classification effect by assigning weights to the input information and finally summing the weights.

##### 3.1.2.5. Experiments

In our experiments, we divide the dataset into training set, validation set and test set in the ratio of 6:2:2. The TextCNN and BiLSTM-Attention models utilized the Adam optimizer, an initial learning rate of 0.001, a batch size of 128, and the probability of dropout of 0.5. This task adopts the CrossEntropy Loss function, which minimizes the cross entropy of the predicted and true results so that they are as similar as possible. The loss function is as follows.


(3) $$\begin{array}{l} L=-\frac{1}{N}\underset{i}{\sum }\overset{M}{\underset{c=1}{\sum }}y_{ic}log\left(p_{ic}\right) \end{array}$$

where *N* is the number of samples, *M* is the number of categories, *y*_*ic*_ is the symbolic function, and *p*_*ic*_ is the prediction probability.

We use accuracy as the evaluation metric, and only a sentence that is predicted with the correct label is considered as a correctly classified sample. The results of each model are shown in Table 1.

**Table 1:** Results of sentence classification.

**Model**	**Accuracy**
SVM	0.5163
XGBoost	0.6466
TextCNN	0.7005
BiLSTM-Attention	0.6637

The classification accuracy of the test set shows that the deep learning models are more accurate than the machine learning models, and TextCNN has the best classification of policy text sentences in our data.

Also, there are some useful findings in our labeled dataset. For example, the percentage of contents related to policy tools reached 75.79% of all labels, wherein those related to funding support and object programming accounted for 24.98% and 17.59%, respectively, with the highest percentage. To some extent, it indicates that the governments issuing these policies prefer to use these two categories of policy tools. Furthermore, we can apply our model to more policies in more regions by automated policy sentence classification to efficiently obtain such information from a large number of policy texts.

#### 3.1.3. Policy information retrieval

##### 3.1.3.1. Task description

This task focuses on the automated extraction of basic information from a policy, which helps to automate the analysis of a large number of policies and may also facilitate the fill in of basic information when the government uploads a policy document. The base information contains: policy name, policy document number, target field, policy-making department, policy implementation department, and validity period.

The article "What is policy content and how is the public's policy support? A policy cognition study based on natural language processing and social psychology" was published in 2022. Journal: Front Psychol.

Specifically, the policy information retrieval task is modeled as a fine-grained Named Entity Recognition (NER) task for unstructured text in NLP. Named entities refer to phrases with specific meanings, which are all kinds of basic information of policy. This concept was first proposed in the message understanding conference series (Grishman and Sundheim, 1996) for information extraction. While common named entities generally include names of people, addresses, organization names, etc., we want to recognize the name, document number, issuing area and others. It is actually a fine-grained Named Entity Recognition task.

The basic task of named entity recognition is to predict the classes and boundaries of all entities in the text. During the training process, the model is constantly updated by the loss between the predicted entity information and the real entity information, and finally adjusted to the state with the best prediction. NER is a sequence annotation problem and a generic upstream foundation task for much of the work in natural language processing. However, it is often poorly generalizable, and currently common named entity recognition systems are difficult to apply to our task of retrieving policy information directly from policy texts. Therefore, we employed and compared several models based on deep learning techniques.

Overall, we analyze this task based on deep learning techniques with distributed representation, context encoding and decoding.

##### 3.1.3.2. Distributed representation

In this task, we used both word-level and character-level distributed representations by implementing pre-trained vectors from Word2vec and pre-trained model RoBERTa (Liu et al., 2019), respectively. This pre-trained model is a more finely tuned version of BERT. The pre-trained models can learn extensive knowledge before training, and dynamic pre-trained models such as RoBERTa can be fine-tuned to fit downstream tasks, often improving the efficiency and effectiveness of training. We use the paradigm of pre-training and fine-tuning, with the pre-trained Chinese RoBERTa model (Cui et al., 2020). We fine-tune the model on the training dataset for our downstream policy information retrieval task.

##### 3.1.3.3. Context encoding

The context encoding layer takes over the output of the distributed representation layer and further models the dependencies between text semantics and words. In our experiments, the Multi-Layer Perceptron (MLP), Transformer, and Flat-Lattice Transformer are used for comparison.

The article "What is policy content and how is the public's policy support? A policy cognition study based on natural language processing and social psychology" was published in 2022. Journal: Front Psychol.

The Multi-Layer Perceptron is the simplest fully connected forward neural network. Its basic structure consists of an input layer, several hidden layers, and an output layer. We use a three-layer structure, including a linear input layer, a ReLU layer and a linear output layer.

Transformer was proposed in 2017 (Vaswani et al., 2017), and its core is self-attention mechanism. Transformer captures long-range dependencies in text, which overcomes the imbalance of sentence length and entity length, and it also incorporates location information through positional encoding. Only the Transformer Encoder is needed to model the text features in our context encoding layer.

FLAT (Flat-LAttice Transformer) (Li et al., 2020) is a Transformer variant that was proposed in mid-2020. It uses both distributed representations of characters and words of text, and further extends the location encoding in Transformer. Specifically, the model expands its positional information by using the first and last relative positions of characters and words. This model can help us overcome the problem of entity length imbalance to some extent.

##### 3.1.3.4. Decoding

In the decoding layer, we use a conditional random field (CRF) model. The CRF model is able to learn some constraints from the output of the previous layer, which makes it more likely to recognize the correct decoded sequence of tags. The decoding process uses the Viterbi algorithm (Forney, 1973), a dynamic planning method, in order to achieve high decoding efficiency.

##### 3.1.3.5. Experiments

In the experiments of this task, we use the BIO^2^ strategy to tag the entities in the sentence sequence and similarly divide the dataset into a training set, a validation set and a test set in the ratio of 6:2:2. The models for entity recognition utilized the Adam optimizer, a batch size of 64, and the probability of dropout of 0.5. For the initial learning rate, it is set to 0.00003 for the pre-trained model part, 0.005 for the conditional random field part, and 0.01 for the other parts.

We use a conditional random field loss function in our training and maximize the conditional probability of predicting the correct label sequence. The expression for the loss is as follows:


(4) $$\begin{array}{l} \;s(x,y)=\sum_{i=0}^{n}T_{y_{i},y_{i+1}}+\sum_{i=0}^{n}E_{i,y_{i}}\\ p(y_{gold}|x)=\frac{e^{s(x,y_{gold})}}{\sum_{y\in Y_{x}}e^{s(x,y)}}\\ \;Loss=-log[p(y_{gold}|x)] \end{array}$$

where *T* is the transfer matrix, *E* is the emission matrix, *x* is the observed sequence, *y*_*i*_ is the *i*-th time step of the label sequence *y*, *y*_*gold*_ is the correct sequence and *s* is the score of each sequence. The purpose of the loss function is to maximize the probability that the model predicts the correct sequence, which means maximizing *p*(*y*_*gold*_|*x*).

The article "What is policy content and how is the public's policy support? A policy cognition study based on natural language processing and social psychology" was published in 2022. Journal: Front Psychol.

The evaluation metrics are Precision (P), Recall (R) and F1-score. These metrics are calculated as follows, where TP is the number of positive cases predicted correctly, FP is the number of negative cases predicted incorrectly, TN is the number of negative cases predicted correctly, and FN is the number of positive cases predicted incorrectly. We use micro-F1 for our multi-classification problem.


(5) $$\begin{array}{l} \begin{array}{c} \;P=\frac{TP}{TP+FP}\\ \;R=\frac{TP}{TP+FN}\\ F1=\frac{2*P*R}{P+R} \end{array} \end{array}$$

The results of each model are shown in Table 2.

**Table 2:** Results of entity recognition.

**Model**	**P**	**R**	**F1**
RoBerta + MLP + CRF	0.6691	0.6852	0.6635
RoBerta + Transformer + CRF	0.5813	0.6629	0.6113
RoBerta + FLAT + CRF	0.7182	0.6977	0.6944

The performance of each model in policy information retrieval shows that the model based on named entity recognition technology can extract the basic information of policy text well. And adding more text information, especially location information, to the extracted features can significantly improve the extraction effect. After achieving efficient automated policy information extraction, the model can be used for larger scale policy text data and for further applications as filtering policies based on the selection of information.

### 3.2. Policy support analysis

#### 3.2.1. Research design

##### 3.2.1.1. Sampling and data collection

We conducted an online survey with the target audience of employees from the whole country and different industries in April 2022. The data is collected by a professional questionnaire survey company, Wenjuanxing, and the respondents' concentration is guaranteed through attention test^3^ during the process. According to the pilot survey, the normal answering time is more than 3 minutes. Thus, we dropped the questionnaires if the answering time was less than 3 minutes in the online survey. Finally, we had 476 valid questionnaires from 22 provinces and 16 industries.

As shown in Table 3, 39.29% of the respondents are male and 60.71% are female, with an average age of 29.3 years old. Also, 348 respondents (73.11%) hold a college degree and 58 (12.18%) hold a postgraduate degree or higher. Most of the respondents' monthly incomes, measured in yuan (RMB), ranges from 5,000 to 10,000, which is consistent with the average monthly income of 6027 yuan (RMB) in urban China in 2020^4^. In terms of position rank, over 70% of respondents are the general staff in their companies, while 27.73% is middle-level leader and only 1.68% is senior leaders. Additionally, 130 respondents are members of the Communist Party of China, and 38.24% works in government agencies or state-owned enterprises while 50.84% works in private enterprises. At last, most respondents' enterprises are medium size, accounting for 35.5%, and 30.46% works in small companies. Generally, our sample is representative of the employees in our country as a whole.

The article "What is policy content and how is the public's policy support? A policy cognition study based on natural language processing and social psychology" was published in 2022. Journal: Front Psychol.

**Table 3:** Distribution of samples.

**Characteristics**		**Frequency**	**Percentage (%)**
Gender	Male	187	39.29
	Female	289	60.71
Age	18–29	304	63.87
	30–39	144	30.25
	40–49	22	4.62
	50–59	6	1.26
	>60	0	0
Education	Middle school or below	2	0.42
	High school	68	14.28
	College	348	73.11
	Master's or above	58	12.18
Monthly income	<3,000	9	1.89
	3,000–5,000	65	13.66
	5,001–8,000	175	36.76
	8,001–10,000	119	25
	>10,000	108	22.69
Job rank	General employees	336	70.59
	Mid-level management	132	27.73
	High-level management	8	1.68
Political background	Communist party member	130	27.31
	Others	346	72.69
Type of working enterprise	Government agencies and state-owned enterprises	182	38.24
	Private enterprises	242	50.84
	Others	52	10.92
Enterprise size	Large	123	25.84
	Medium	169	35.5
	Small	145	30.46
	Micro	39	8.19

##### 3.2.1.2. Measurement design

We designed the questionnaire in five sections, measuring policy support for supply, demand and environmental tools, political trust, policy effectiveness, knowledge of policies and socio-demographic characteristics. Except for socio-demographic variables, other parts are all in the form of Likert's five-point scale, where “1” means strongly disagree, “3” means neutral, and “5” means strongly agree.

*Policy support*, the dependent variable, is measured directly by the degree of support for a certain policy tool. In the questionnaire, we asked the respondent to choose how much they support with policy tools as personnel training, financial support, technical support and others. As listed in 3.1.1, there are totally 13 tools, including 4 supply tools, 3 demand tools and 6 environmental tools.

For independent variables, we try to measure *political trust* more comprehensively rather than a single question as “how much do you trust in the government generally”. In this paper, this concept is captured from how much the respondents agree with five statements: “I believe that the government's decision-making represents the public interest”, “I believe that the policy-making process of government agencies is open and transparent”, “I think I have the capacity to participate in the policy making process”, “I believe that the government is capable to support the development of enterprises”, “I believe that the government is capable to promote economic development”.

The article "What is policy content and how is the public's policy support? A policy cognition study based on natural language processing and social psychology" was published in 2022. Journal: Front Psychol.

Additionally, *policy effectiveness* refers to how well the social effect could be generated by the implementation of certain policies. Our paper measures policy effectiveness subjectively by asking the respondents how effective they think about different policy tools. Similarly, we capture the respondents' *knowledge of policies* from their self-reported judgement, by asking “How well do you know the following policies?”.

Besides age, gender, education, income, we also test whether the respondents are party member, their position rank, working years and the details of working enterprise including size and ownership.

In terms of scale reliability, we test Cronbach's α value, the average linear correlation among questions belonging to the same scale. According to Hinton et al. (2014), “…0.5 to 0.75 is generally accepted as indicating a moderately reliable scale, while a figure below this generally indicates a scale of low reliability”. In our paper, the Cronbach's α values of policy support, policy effectiveness and knowledge of policies are all over 0.8, and that of political trust is over 0.6 as shown in Table 4. Therefore, our scale can be considered as reliable.

**Table 4:** Reliability test over the measurements.

**Variable**	**Cronbach's α**	**The number of items**
Policy support	0.8317	13
Political trust	0.6308	5
Policy effectiveness	0.8948	13
Knowledge of policies	0.8870	13

#### 3.2.2. Empirical results

##### 3.2.2.1. Descriptive comparison of supply, demand, and environmental tools

First, we conducted a descriptive statistical analysis to compare the variables of policy support, policy effectiveness, knowledge among supply, demand and environmental tools and political trust. As shown in Table 5, regarding policy support, most respondents support for these policy tools, especially for supply tools, with the mean of 4.24. This result indicates that the audience prefer supply tools such as talent training, technical or financial support and others. Additionally, we find that compared with demand and environmental tools, respondents think the supply tools are most effective and have the highest level of knowledge about this tool. In that sense, we could attribute the audience' highest level of support for the supply tool to its effectiveness and relevant knowledge. Lastly, the mean of political trust is 3.98, and more than 75% respondents trust in the governmental agencies' willingness and capacity to promote economic development and enhance enterprise success.

The article "What is policy content and how is the public's policy support? A policy cognition study based on natural language processing and social psychology" was published in 2022. Journal: Front Psychol.

**Table 5:** Distribution of key variables for the three policy tools.

		**Supply tools**			**Demand tools**			**Environmental tools**		
		**Dist. (%)**	**Ave**.	**S.D**.	**Dist. (%)**	**Ave**.	**S.D**.	**Dist. (%)**	**Ave**.	**S.D**.
Policy support	Disagree	2.2	4.24	0.75	4.62	3.99	0.86	3.71	4.11	0.82
	Neutral	11.34			21.15			16.46		
	Agree	86.45			74.23			79.83		
Policy effectiveness	Disagree	16.65	3.53	1.02	23.81	3.30	1.09	17.82	3.5	1.04
	Neutral	29.2			30.88			29.59		
	Agree	54.15			45.31			52.59		
Knowledge of policies	Disagree	15.97	3.59	0.99	26.19	3.30	1.09	17.4	3.55	1.02
	Neutral	22.48			23.81			22.93		
	Agree	61.55			50			59.66		
Political trust	Disagree	8.15							3.98	0.95
	Neutral	16.47								
	Agree	75.38								

Political trust represents the public's judgment of the government, and it does not vary based on policy tools.

##### 3.2.2.2. Analysis of the influencing factors of policy support

To better delineate the formation mechanism of policy support, we try to further analyze the influencing factors of policy support. As shown in model (6), this paper takes “policy support” as the dependent variable and political trust, policy effectiveness and knowledge of policies as well as socio-demographics as independent variables (*X*_*i*_) for regression analysis. We adopt the ordinary least square (OLS) method to analyze the data.


(6) $$\begin{array}{l} Policy\;support=\alpha +\beta X_{i}+u \end{array}$$

First, we do a confirmatory factor analysis for policy support, policy effectiveness and knowledge of polices for supply, demand and environmental tools, and political trust to reduce the dimensions and combine them into one factor separately. The coefficients of Kaiser-Meyer-Olkin test are shown in Table 6. All of them are above 0.6, indicating that they are suitable for factor analysis. Then, we run the model (6) and finally get the regression results as shown in Table 7.

**Table 6:** Kaiser-Meyer-Olkin test of key variables.

**Variables**		**Coefficient of KMO test**	**The number of items**
Policy support	Supply tools	0.7077	4
	Demand tools	0.6220	3
	Environmental tools	0.7099	6
Political trust		0.7215	5
Policy effectiveness	Supply tools	0.7656	4
	Demand tools	0.6777	3
	Environmental tools	0.8114	6
Knowledge of policies	Supply tools	0.7790	4
	Demand tools	0.6804	3
	Environmental tools	0.7797	6

**Table 7:** Influencing factors of policy support.

	**Support_Whole Sample**		**Support_Supply**		**Support_Demand**		**Support_Environment**	
	**Coef**.	**S.E**.	**Coef**.	**S.E**.	**Coef**.	**S.E**.	**Coef**.	**S.E**.
Political Trust	0.57^****^	0.047	0.46^****^	0.042	0.27^****^	0.037	0.40^****^	0.043
Policy Effectiveness	0.19^****^	0.046	0.14^***^	0.044	0.21^****^	0.042	0.24^****^	0.043
Knowledge of policies	–0.17	0.045	–0.07^*^	0.042	0.08^**^	0.042	0.05	0.043
Gender	0.04	0.072	0.06	0.064	0.02	0.059	0.04	0.066
Age	0.11	0.069	0.04	0.061	0.08	0.056	0.13^**^	0.063
Education	0.08	0.065	0.08	0.058	–0.05	0.053	0.12^**^	0.060
Income	0.13^***^	0.039	0.11^***^	0.035	0.05^*^	0.032	0.10^***^	0.036
Political Background	–0.06	0.082	0.01	0.073	–0.08	0.068	–0.10	0.076
Job Rank	0.01	0.075	–0.01	0.067	0.09	0.062	–0.03	0.069
Working Year	–0.01	0.011	–0.006	0.010	–0.007	0.009	–0.01	0.010
Enterprise size	0.001	0.042	0.03	0.037	0.02	0.034	–0.04	0.038
Type of working enterprise	–0.09	0.077	–0.06	0.069	–0.05	0.063	–0.09	0.070
*R* ^2^	0.3780		0.3165		0.2716		0.3405	
*N*	476		476		476		476	

* *p* < 0.1,

** *p* < 0.05,

*** *p* < 0.01,

**** *p* < 0.001.

The article "What is policy content and how is the public's policy support? A policy cognition study based on natural language processing and social psychology" was published in 2022. Journal: Front Psychol.

First, the employees who trust more in governments tend to have higher level of support for all policies (β = 0.57, *p* < 0.001). Especially, the significant and positive effect of political trust is strongest in the sample of supply tool (β = 0.46, *p* < 0.001), while weakest in the sample of demand tool (β = 0.27, *p* < 0.001). This result is consistent with exiting studies, verifying the positive correlation between political trust and policy support. The audience are more likely to abide by the decisions of political agencies if they trust in and perceive these agencies as legitimate (Tyler and Huo, 2002).

Second, the more the employees perceive policies as effective, the higher they support these policies (β = 0.19, *p* < 0.001). This positive relationship is more obvious for environmental tools, with a β coefficient of 0.24 and a *p*-value less than 0.001. Scholars found that policy effectiveness has positive effects on the public's support for certain policies (Zannakis et al., 2015). We believe that the audience would perceive more benefits of policies when they are regarded as effective, and tend to be more willing to support these policies.

Additionally, knowledge of policies has different effects on the employees' support for supply, demand and environmental tools. Specifically, for supply policy tool, people with more knowledge tend to be less likely to support them (β = −0.07, *p* < 0.1), while the relationship changes to a positive one in the sample of demand tool (β = 0.08, *p* < 0.05). And knowledge of polices does not show any significant effects for the environment tool. These inconsistent results may be related to the respondents' knowledge content and the characteristics of different policy tools. Also, there might be a bias about self-reported knowledge level, which has been stated in existing literature (Costa-Font et al., 2008). Further exploration is needed to figure out the relationship and causal mechanism between knowledge and policy support for different tools.

The article "What is policy content and how is the public's policy support? A policy cognition study based on natural language processing and social psychology" was published in 2022. Journal: Front Psychol.

As last, among the socio-demographic factors, income has a positive and significant effect on policy support for the whole (β = 0.13, *p* < 0.01) and this impact also exist for each policy tool. Typically, the employees with higher income might be the group that benefit more from policies, thus they are more willing to support these policies.

## 4. Conclusion and discussion

Policy documents are important action guidelines and strategies for governments to coordinate resources and provide social services, and the public might have different policy cognition objectively and subjectively. It's of great significance for us to explore both the content and support of policies, which is beneficial to policy legitimacy and implementation. Therefore, the first part of our paper analyzed the policy text automatically by deep learning and machine learning methods after establishing a system of policy elements. Then we analyzed the key factors on policy support for supply, demand and environmental tools in three dimensions: political trust, policy effectiveness and knowledge of policies.

The results of the experiments based on policy text showed that the deep learning models could achieve better results for the policy content analysis than the machine learning models. We also found that the model extracting text features spatially achieved better results than the model extracting text features temporally. This might be because of the characteristics of policy text in the dataset. Additionally, as the entity length of the policy text tends to be long, increasing the information in the location encoding can improve the model considerably. By automating the classification of policy sentences and the identification of policy information, it is possible to parse large amounts of policy texts with great efficiency. In terms of specific applications, policy tools, namely supply, demand and environmental tools, distinguished by the classifier can be used to analyze the main content of policy documents. It is also possible to extract structured information related to specific policies from documents quickly through the policy information identification task, which can be applied to filter out policy-related departments, enterprises and other subjects.

In the study of policy support analysis, we employed the factor analysis and ordinary least square method to analyze the influencing factors of policy support. First, political trust and policy effectiveness have positive effects on policy support. Citizen's trust in governments, meanwhile, represents their belief that the government is able to formulate effective policies and implement them correctly, so they are more supportive for the policies designated by the government. The government could enhance the support of policy tools via improving policy effectiveness and facilitating political trust. On the one hand, the government should devote more resources to existing policies and launch more effective policy tools according to the practical situation. On the other hand, putting the public back into the policy-making process can promote the transparency of policy-making and enhance citizens' trust in governmental agencies.

The article "What is policy content and how is the public's policy support? A policy cognition study based on natural language processing and social psychology" was published in 2022. Journal: Front Psychol.

However, this study also has some limitations. First, most of the policy document data used for policy text analysis are published by Zhejiang Province. The lack of samples from other provinces poses a challenge to the external validity of our results to some extent due to the different economic situations and development strategies of each region. Second, the structure of the neural network used in this study is relatively simple, and its performance in specific tasks can be further improved. Third, in the policy support study, questionnaires are subjective “self-reports” of respondents, which might inevitably deviate from their real behavior. In addition, as people are highly likely to overestimate their abilities in self-reported assessment, our self-rated measurement of knowledge might generate threats to validity and reliability. Fourth, the study found that the influencing factors of different policy tools are slightly different, but the existing data cannot explain these differences in detail. Usually, the results obtained from statistical regression require further supplementation and explanation by qualitative research.

## Data availability statement

Requests to access these datasets on which this article is based should be directed to SC, simingchen3@gmail.com.

## Author contributions

LZ: framing the paper, study design, discussion, and writing. DD: implement the work, conducting user study, writing, and discussion. XC and JR: data provider, discussion, expert study, and proofreading. SC: framing the paper, discussion, writing, and evaluation. All authors contributed to the article and approved the submitted version.

## Funding

This work was funded by Shanghai Pujiang Program (Grant/Award No. 2020PJC018), Shanghai Municipal Science and Technology Major Project (Nos. 2018SHZDZX01 and 2021SHZDZX0103), General Program (No. 21ZR1403300), Sailing Program (No. 21YF1402900), and ZJLab (NSFC No. 62202105).

The article "What is policy content and how is the public's policy support? A policy cognition study based on natural language processing and social psychology" was published in 2022. Journal: Front Psychol.

## Conflict of interest

Author JR was employed by Tiandao Fintech Co., Ltd., Hangzhou, China and Author XC was employed by Zhelixin Co., Ltd., Hangzhou, China.

The remaining authors declare that the research was conducted in the absence of any commercial or financial relationships that could be construed as a potential conflict of interest.

## Publisher's note

All claims expressed in this article are solely those of the authors and do not necessarily represent those of their affiliated organizations, or those of the publisher, the editors and the reviewers. Any product that may be evaluated in this article, or claim that may be made by its manufacturer, is not guaranteed or endorsed by the publisher.

## Footnotes

^1^ https://www.zj.gov.cn/col/col1229614259/index.html

^2^We use B, I, O and entity type to mark the beginning words of the entity, the middle words of the entity, and the words that are not part of the entity.

^3^E.g., “When I'm not working, I'll travel on the moon”, “Where is the capital of China?”

^4^Released by the National Bureau of Statistics in 2021. http://www.stats.gov.cn/tjsj/ndsj/2021/indexch.htm.
